# The optimization of the "UAV-vehicle" joint delivery route considering mountainous cities

**DOI:** 10.1371/journal.pone.0265518

**Published:** 2022-03-21

**Authors:** Wusheng Liu, Wang Li, Qing Zhou, Qian Die, Yan Yang

**Affiliations:** 1 Engineering Research Center of Catastrophic Prophylaxis and Treatment of Road & Traffic Safety of Ministry of Education, Changsha University of Science & Technology, Changsha, Hunan, China; 2 School of Traffic and Transportation Engineering, Changsha University of Science and Technology, Changsha, China; Southwest Jiaotong University, CHINA

## Abstract

As a new transportation tool, unmanned aerial vehicle (UAV), has a broad application prospect in logistics distribution, especially for mountainous cities with complex terrain. Due to the limited delivery conditions of UAV, considering the advantages of traditional vehicle delivery, this paper proposes a joint delivery mode of UAV and vehicle, and designs three steps for the joint delivery problem of single UAV and single vehicle: first, mark all special nodes; Secondly, the route of UAV and vehicle is planned; Finally, the total delivery route is optimized to minimize the total delivery distance. Genetic algorithm and single distribution terminal optimization are used to solve the problem, and the joint delivery in this paper is compared with the traditional vehicle delivery and the independent delivery of UAV and vehicle. The results show that UAV and vehicle can cooperate with each other to complete the delivery of all customer demand nodes, and the joint delivery of UAV and vehicle can effectively reduce the total delivery distance. Finally, the sensitivity analysis of UAV’s maximum load, maximum flight distance, relative speed between UAV and vehicle, and road impedance coefficient is carried out. By relaxing the restrictions of UAV, the UAV can deliver more customers at a single time, and it complete the delivery task with vehicles efficiently.

## 1 Introduction

With the continuous development of e-commerce, enterprises and customers have been seeking faster and more efficient logistics. However, in mountainous cities with complex terrain and poor traffic conditions, logistics distribution is often hindered by mountains and rivers. How to effectively complete the "last mile" delivery is an urgent problem to be solved. The civil UAV provides a new solution to this problem.

At first, UAV (Unmanned Aerial Vehicle, or Drone) was mainly used for coordinated operations in the military field [1]. In recent years, civilian UAVs have developed rapidly. With their advantages of convenient operation, flexible use, high operating efficiency, and low relative cost [2], the application scope has been expanded to logistics distribution, surveillance cruise, emergency rescue, and medical transportation [3–7]. However, due to the small load capacity and the inability to support long-distance flights, there are many restrictions in the delivery of goods. Traditional delivery vehicles have the advantages of large load capacity and long-distance transportation. The combined delivery potential of the two is huge. It has become one of the research hotspots in recent years.

Wohlsen et al. [8] first proposed the use of trucks and UAVs for collaborative cargo delivery. In this problem, the truck and the UAV can deliver to customers independently, but the UAV needs to return to the truck to take a package after each delivery. From this idea, Agatz et al. [9, 10] called this path problem as the traveling salesman problem with drone (TSP-D), with the goal of minimizing delivery costs, and constructed a mixed integer model of TSP-D. Ha et al. [11] aimed at the TSP-D problem of single truck and single UAV, aimed at minimizing the total delivery cost and the penalty cost of truck waiting for UAV.

In addition, Murray et al. [12] proposed the flying sidekick traveling salesman problem (FSTSP) and the parallel drone scheduling traveling salesman problem (PDSTSP) two models for the coordinated delivery of UAVs and trucks, with the goal of minimizing service time. Yurek et al. [13] designed a two-stage iterative algorithm for solving FSTSP and compared it with the solution time of CPLEX, the results showed that the algorithm can reduce the solution time for medium-scale examples. Ham [14] extended PDSTSP, taking into account that UAVs can pick up or deliver goods at warehouses or customer locations at the same time, and use multi-truck, multi-UAV and multi-warehouse joint delivery problems to verify.

The above studies all proceed from the TSP problem, assuming that a single UAV launch can only serve one customer, and the vehicle launches and receives the UAV at a fixed point. However, these assumptions impose a lot of restrictions on joint delivery. The research of Bouman et al. [15] also shows that the number of nodes that the UAV can visit when leaving the truck can significantly shorten the total delivery time. UAVs should be allowed to deliver multiple packages within a reasonable tolerance range. In addition, the sending and receiving of UAVs by vehicles can be a dynamic process, which can give greater play to the mobility of joint delivery. This paper has also made improvements in these aspects.

In terms of improving the efficiency of joint delivery, Savuran et al. [16] proposed a new variant of MoDVRP (Mobile Depot VRP), he assumes that the vehicle is moving along a straight line, with a large number of customer points delivery on both sides of the route, and that as many customer points are delivered as possible after the UAV takes off. Regarding the limitation of UAVs, Wang et al. [17] considered the UAV vehicle path problem VRP-D under the limitation of endurance, for the coordinated delivery of multiple trucks and UAV, it is proposed that UAVs can be launched and received from trucks in warehouses or any customer location. Dorling [18] considered the relationship between the flight distance and load of the UAV, and concluded that energy consumption and delivery time cannot be optimized at the same time. In order to effectively solve the VRP-D problem, Scherme et al. [19] found the optimal allocation and scheduling of UAVs based on a mixed integer linear programming model.

Considering the complexity of the joint delivery problem of vehicles and UAVs, researchers can simplify the solution process, and the solution ideas can be divided into the following two categories. One is based on routing first [8, 9], that is, to solve the truck route according to the traditional TSP problem, and then to allocate the UAV route according to the priority criterion, and to optimize the final route allocation by the objective function; the other is based on clustering first [12], that is, to calculate the cluster centers from the customer distribution characteristics, the truck is responsible for the delivery of each center point, and then allocate the driving route of trucks, deliver to the surrounding customer points.

All these studies have the same steps: determine the route of the truck first, and then allocate the flight route of the UAV, and use the idea of gradual approximation [20] and classification [21] to design heuristic algorithm to solve the joint delivery problem. Generally, the designed heuristic algorithm can get better results, but it can only solve small-scale cases, and the calculation time is very long [14] (Solving 10 customer cases takes more than one hour). In order to make the solution more efficient, researchers began to use meta heuristic algorithm to improve the operation efficiency, such as Simulated Annealing Algorithm [19], Greedy Algorithm [12], Neighborhood Search Algorithm [22], etc., which makes the joint delivery problem can be extended to large-scale cases, while greatly reducing the operation time and gaining better results. But in general, this kind of research is still not taken widely. This paper attempts to determine the delivery route of UAV first, so that it can serve more customers at a time, and then allocate the driving route of trucks, and designs a genetic algorithm with terminal optimization to solve the proposed joint delivery model.

Compared with vehicle, UAV is faster and more convenient, and the cost is lower. In the future, UAVs will be more widely used in distribution. Researchers have also conducted a large number of studies to confirm the advantages of joint delivery in time [23] and cost [13], but the researchers rarely pays attention to the path distance, especially for complex terrain such as mountains and hills. Due to road bending, large slope and ups and downs, traditional vehicle delivery is very inconvenient, and the utility of time and cost is relatively low. In some areas surrounded by hills and lakes, vehicles cannot be delivered at all, and UAV delivery is not affected by terrain, which greatly shortens the delivery distance, and UAV delivery has great advantages in areas where mountains and rivers are blocked and vehicles cannot enter.

Considering that most nodes in mountainous cities are clustered and distributed in blocks, and there are many special customer points. In order to complete the "last mile" delivery, the main contributions of this paper are as follows:

1. Based on the scenario of single UAV and single vehicle, this paper constructs the UAV-vehicle joint delivery model, reasonably plans the delivery of special points, and arranges as many customer points as possible to UAVs;
2. Under the limitation of load and flight distance, the UAV can deliver multiple packages at a time. The vehicle can carry the UAV for delivery, and can also deliver with the UAV at the same time. The two cooperate to complete the delivery task together.
3. Aiming at the shortest delivery route, a heuristic algorithm is designed to solve the model, and the results are compared with other scenarios to verify the feasibility of the model.

The rest of this paper is arranged as follows: in Section 2, the problem is described in detail, and the definition and hypothesis of the problem are also given. In sections 3 and 4, the model and algorithm designed in this paper are given respectively, which is applied to solve problem in Section 5. We also make sensitivity analysis on several parameters to obtain a more comprehensive understanding. The conclusion is in Section 6.

## 2 Problem description

Due to the distribution advantages of UAVs, large logistics enterprises such as Amazon, DHL and JD have increased the experiment of UAV delivery. As a new transportation tool in logistics distribution, UAV has the advantages of low cost, convenient operation, low environmental requirements and strong survivability. It has great potential in logistics transportation application and can undertake more delivery tasks. However, because of its small volume, small load capacity, short flight distance and great influence by the weather, the traditional delivery vehicle has the advantages of large capacity, long-distance delivery, high safety and stability and mature related distribution technology. The joint delivery of UAV and vehicle can give full play to their respective advantages.

This paper gives the following definitions:

1. Vehicles: including trucks, tricycles and other means of transport that can distribute goods and support UAV launch and return.
2. Impedance: it is not limited to the non-linear coefficient, slope, flatness of the road, and other factors that can affect the smooth and uniform driving of vehicles.
3. Joint delivery: the UAV needs to pick up the goods from the vehicle and return to the vehicle after the delivery. The vehicle can carry the UAV for delivery, and can also simultaneously carry out the delivery of other customer points after the UAV picks up the goods. The two cooperate to complete the delivery of all customer points according to the specific characteristics of the customer points.
4. Independent delivery: that is, non-joint delivery, vehicles and UAVs independently to complete their own delivery tasks.
5. Docking point: it can be used for vehicles to park and wait for UAV, where UAV can complete battery replacement, goods removal, or launch recovery. The docking point can be any customer point or delivery center.

A simple mode of UAV vehicle joint delivery studied in this paper is shown in Fig 1. In the figure, UAVs and vehicles can respectively carry goods out of the delivery center, or vehicles can carry UAVs back to the delivery center; When the UAV is delivering, the vehicle doesn’t have to stay in the place and wait, but can deliver at the same time. A single distribution of UAV can serve multiple customer points at the same time. In addition, the super far nodes exceeding the maximum flight distance of the UAV are marked in red in the figure. Because the UAV cannot go back and forth for a long distance, the super far customer nodes can only be delivered by vehicles. The overweight nodes can only be delivered by vehicles because the UAV can’t load heavy goods, but the UAV can fly to the overweight nodes for parking.

**Fig 1:** Joint delivery of single UAV and single vehicle.

The three service forms of overweight node are shown in Fig 2: in figure (a), overweight node can be used as the parking point of UAV and vehicle; In figure (b), the vehicle can carry UAV to distribute the overweight nodes; In figure (c), both UAVs and vehicles distribute to customer points, and the vehicle is responsible for the overweight nodes.

**Fig 2:** The overweight node service form.

Based on the above problems, this paper makes the following assumptions

1. The location and demand of delivery center and customer point are known, and the demand of delivery center is 0;
2. All customer points must be served, regardless of the time window of customer points;
3. The maximum load and range of UAV are known;
4. The UAV can serve more than one customer point at a time under the limited conditions;
5. Regardless of the load limit and endurance limit of the vehicle;
6. The vehicle must arrive at the stop before the UAV, and the UAV cannot hover at the stop;
7. After each delivery, the UAV needs to return to the vehicle to pick up the goods and replace the battery;
8. The service time of the customer point and the time of UAV picking up and battery replacement are not considered;
9. Enough UAV power supply is carried on the vehicle.

## 3 Mathematical model of joint delivery

### 3.1 Parameter description

The parameters used in the modeling process are as follows:

***S***: The set of all nodes, ***S*** = {1, 2, ⋯, *n*, *n* + 1}, Where *n* + 1 is the delivery center;
***C***: The set of all customer demand nodes, ***C*** = {1, 2, ⋯, *n*};
***N***: The set of customer demand nodes not served, ***N*** = {1, 2, ⋯, *n*};
***R***_***m***_: The set of customer demand nodes exceeding the maximum load limit of UAV;
***R***_***d***_: Customer demand nodes set whose distance from other customer nodes exceeds the maximum flight distance limit of UAV;
***U***: The set of customer demand nodes for UAV delivery, ***U*** = {***U***_**1**_, ***U***_**2**_, ⋯, ***U***_***k***_};
***U***_***k***_: Customer demand point set of UAV delivery for the kth distribution;
***T***: The set of customer demand nodes for Vehicle delivery, ***T*** = {***T***_**1**_, ***T***_**2**_, ⋯, ***T***_***k***_};
***T***_***k***_: Customer demand point set of Vehicle delivery for the kth distribution;
***P***: The set of all parking spots;
***K***: Total number of distribution, ***K*** = {,1 2, ⋯, *k*};
*n*: Total number of customer demand nodes;
|*U*_*k*_|: Customer demand points of UAV delivery for the kth distribution;
|*T*_*k*_|: Customer demand points of Vehicle delivery for the kth distribution;
*m*_*i*_: Cargo demand of node i;
*d*_*ij*_: Euclidean distance from node i to node j;
*M*: Maximum payload of UAV;
*D*: The maximum flight distance of UAV;
*v*_1_: Average flight speed of UAV;
*v*_2_: Average speed of vehicle;
*ε*: Road impedance coefficient;
*E*_*k*_: The sum of the distances of the UAV delivery routes for the kth distribution;
*F*_*k*_: The sum of the distances of the vehicle delivery routes for the kth distribution;
*Z*: Total mileage of delivery routes;

xij,k=1,Atthekthdistribution,theUAVmovesfromnodeitonodej0,Atthekthdistribution,theUAVdidnotmovesfromnodeitonodej

yij,k=1,Atthekthdistribution,thevehiclemovesfromnodeitonodej0,Atthekthdistribution,thevehicledidnotmovesfromnodeitonodej

### 3.2 Model building

In order to minimize the total delivery distance, this paper is divided into the following three steps.

#### (1) Step1: Marking special points

For all demand nodes can be delivered, and the UAV has the maximum load limit and the maximum flight distance limit in a single flight, the demand nodes exceeding the maximum load limit of the UAV are marked as ***R***_***m***_, and the demand nodes exceeding the maximum flight distance limit of the UAV are marked as *R*_*d*_. All marked nodes can only be delivered by vehicles. However, the customer demand nodes marked with *R*_*m*_ can be regarded as the single destination of UAV under the condition of meeting the flight distance limit of UAV.


∑k∈K∑i∈Si≠jyij,k=1∀j∈Rm⋃Rd (1)

∑k∈K∑j∈Si≠jyij,k=1∀i∈Rm⋃Rd (2)

∑k∈K∑i∈Si≠jxij,k=0∀j∈Rd (3)

∑k∈K∑j∈Si≠jxij,k=0∀i∈Rd (4)

0<∑k∈K∑j∈Cj≠i(xij,k+yij,k)≤2i=n+1 (5)

0<∑k∈K∑i∈Ci≠j(xij,k+yij,k)≤2j=n+1 (6)

$$\left|T_{k}\right|\geq 1\forall k\in K$$ (7)

Formula (1) and formula (2) indicate that the marked nodes must be delivered by vehicles; Formulas (3) and (4) denote those nodes marked *R*_*d*_ will not be delivered by UAV; Formula (5) and formula (6) indicate that UAVs and vehicles can enter and exit from the delivery center alone or together with vehicles; Formula (7) shows that each delivery serves at least one customer node.

#### (2) Step 2: Planning single path

*① UAV route*. Due to the limitation of UAV’s power, under the condition that UAV can reach the farthest flight distance radius and meet the maximum load limit of UAV, it is necessary to allocate as many customer demand nodes as possible to UAV. For a given flight radius, the maximum number of customer nodes that UAV can serve in a single distribution is limited. After each assignment, the destination of the single arrival is recorded.


max∑i∈Ni≠j∑j∈Nxij,kk∈K (8)

∑i∈Ni≠j∑j∈Nxij,kmi≤M∀k∈K (9)

∑i∈Ni≠j∑j∈Nxij,kdij≤D∀k∈K (10)

∑i∈Ni≠jxij,k≤1∀j∈N,k∈K (11)

∑j∈Ni≠jxij,k≤1∀i∈N,k∈K (12)

$$N=N-U_{k}\;\forall k\in K$$ (13)

Formula (8) is to maximize the number of customer nodes in a single UAV service; Formula (9) ensures that the cargo weight carried by the UAV in a single time does not exceed the maximum capacity of the UAV; Formula (10) defines that the total delivery distance of a single UAV does not exceed the maximum flight distance of the UAV; Formula (11) indicates that in all unserved customer nodes, the UAV enters the node no more than once; Similarly, formula (12) indicates that the UAV does leaves the node no more than once; Formula (13) that if the customer node of UAV service is allocated, it will be removed from the previous customer node set.

*② Vehicle route*. UAV can not fly for a long time, and carry a limited amount of goods. The vehicle is a mobile station to provide power and goods. Considering the safety, in order to ensure the normal launch and reception of UAV, the vehicle must arrive at the stop before receiving UAV. Taking the end point of the UAV single path planning record as the end point of the vehicle delivery, on the premise of meeting the early arrival, as much as possible to assign customer demand nodes to the vehicle. Due to the limitation of delivery time, the number of customers that can be served by a single vehicle delivery is limited.


max∑i∈Ni≠j∑j∈Nyij,k∀k∈K (14)

εv2∑i∈Ni≠j∑j∈Nyij,kdij≤1v1∑i∈Ni≠j∑j∈Nxij,kdij∀k∈K (15)

∑i∈Ni≠jyij,k≤1∀j∈N,k∈K (16)

∑j∈Ni≠jyij,k≤1∀i∈N,k∈K (17)

$$N=N-T_{k}\;\forall k\in K$$ (18)

Formula (14) is to maximize the number of customer nodes in a single vehicle service; Formula (15) ensures that the vehicle must arrive before the UAV arrives; Formula (16) means that the vehicle does not enter the node more than once among all the customer nodes which are not served; Similarly, formula (17) indicates that the vehicle leaves the node more than once; Formula (18) ensures that every time the customer node of vehicle delivery is allocated, it is removed from the previous customer node set.

#### (3) Step 3: Optimizing the overall route

Take the end point of single distribution route record as the starting point of next distribution route, and repeating the step 2 until all customer demand nodes are delivered. The delivery distance of vehicle and UAV is added, and the shortest total delivery distance is taken as the objective function to optimize the route selection of each delivery.


minZ=∑k∈K∑i∈Si≠j∑j∈S(xij,kdij+εyij,kdij) (19)

∑k∈K∑i∈(S-P)i≠j(xij,k+yij,k)=1∀j∈(S-P) (20)

∑k∈K∑j∈(S-P)i≠j(xij,k+yij,k)=1∀i∈(S-P) (21)

∑k∈K∑i∈(S-P)i≠lxil,k=∑k∈K∑j∈(S-P)l≠jxlj,k∀l∈(S-P) (22)

∑k∈K∑i∈Si≠jyij,k=1∀j∈P (23)

∑k∈K∑j∈Si≠jyij,k=1∀i∈P (24)

∑k∈K∑i∈Si≠lyil,k=∑k∈K∑j∈Sl≠jylj,k∀l∈S (25)

$$x_{ij,k}\in \left\{0,1\right\}\;\forall i\in S,j\in S,k\in K$$ (26)

$$y_{ij,k}\in \{0,1\}\;\forall i\in S,j\in S,k\in K$$ (27)

The objective function (19) is to minimize the total delivery distance between UAV and vehicle; Formulas (20) and (21) indicate that all non parked customer nodes are only delivery once by UAVs or vehicles; Eq (22) ensures the conservation of UAV access flow for non docking points; Formula (23) and formula (24) indicate that vehicles at all stops only enter and exit once; Formula (25) ensures the conservation of vehicle flow in and out for all nodes; Formula (26) and formula (27) give the value range of parameters. Formulas (5), (6) and (20)–(25) jointly give the access rules when the delivery center is used as a stop and non stop, so as to ensure that UAVs and vehicles drive out of the delivery center and finally return to the delivery center without visiting the delivery center again. The pseudo code of formula (8)–(18) is shown in algorithm 1.

Algorithm 1: *Single path planning*()

1 Input: *m*_*i*_, *d*_*ij*_, *M*, *D*, *R*_*d*_, *N* = {1, 2, ⋯, *n*}

2 Output: *U*_*k*_, *T*_*k*_

3 $U_{k}^{*}\leftarrow \emptyset$, $T_{k}^{*}\leftarrow \emptyset$, *m* ← 0, *E_k_* ← 0, *F_k_* ← 0;

4 for *i*, *j* ∈ *N* do

5 *P* ← *P* ∪ {*i*};

6  if *i*, *j* ∈ *R*_*d*_ then

7   continue;

8  else

9   Find *E*_*k*_ + *d*_*ij*_ ≤ *D* in set N;

10   *m* ← *m* + *m*_*i*_;

11   *E*_*k*_ ← *E*_*k*_ + *d*_*ij*_;

12   $U_{k}^{*}\leftarrow U_{k}^{*}\cup \{i\}$;

13   $\left|U_{k}^{*}\right|\leftarrow \left|U_{k}^{*}\right|+1$;

14   if *m* ≥ *M* or constraint (*E*_*k*_ + *d*_*ij*_ ≥ *D*) then

15    *P* ← *P* ∪ {*j*};

16    break;

17   else *i* ← *j*;

18    *j* ← *j* + 1;

19 Repeatedly traverse all nodes n;

20 if $|U_{k}|\leq \left|U_{k}^{*}\right|$ then

21  $U_{k}\leftarrow U_{k}^{*}$;

22 *N* ← *N* − *U*_*k*_;

23 for *l* ∈ *N* do

24  *T*_*k*_ ← *T*_*k*_ ∪ *P*;

25  Optimization of the TSP route, the start and end points are determined by the set P

26  *F_k_* ← *F_k_* + *d_t_star,l_*) + *d_l,t_end_*)

27  $T_{k}^{*}\leftarrow T_{k}^{*}\cup \{l\}$;

28  $\left|T_{k}^{*}\right|\leftarrow \left|T_{k}^{*}\right|+1$;

29  if $\frac{1}{v_{1}}E_{k}\geq \frac{\varepsilon }{v_{2}}F_{k}$ then

30   break;

31 Repeatedly traverse all nodes n;

32 if $|T_{k}|\leq \left|T_{k}^{*}\right|$ then

33  $T_{k}\leftarrow T_{k}^{*}$;

34 *N* ← *N*–*T*_*k*_;

35 return *U*_*k*_, *T*_*k*_;

## 4 Designing algorithm

TSP is a classic NP hard problem. The joint delivery model of single UAV and single vehicle designed in this paper is modified on the basis of Vehicle Routing Problem (VRP), which is different from the capacitated vehicle routing problem (CVRP) and multi types vehicle routing problem (MTVRP), it is the joint delivery problem with both characteristics. Because the complexity of the problem increases exponentially with the number of nodes, this paper uses genetic algorithm to solve the joint delivery routing problem. Genetic algorithm is a heuristic search algorithm based on biological evolution, which can quickly converge to the optimal solution. By setting different genetic operators, it can effectively solve the problem proposed in this paper. The genetic algorithm (GA*) pseudo code designed in this paper is shown in Algorithm 2.

### 4.1 Design of genetic algorithm

#### (1) Chromosome coding

Using integer permutation coding method, the chromosome composed of 1 ~ n integer is randomly generated, each integer gene means n customer demand nodes, and the delivery center is represented by n+1. Each chromosome can be divided into several different parts, and each part is a set of UAVs and vehicle routes with different distribution times. The sequence of each gene determines the delivery order of the corresponding nodes. Starting from the delivery center, each node is added to the delivery route of UAV and vehicle in sequence. Each node is added to calculate whether it meets the constraints. If the constraints are not exceeded, the next node will continue to be added. Until the constraints are exceeded, the next distribution (another vehicle) will be entered. See Algorithm 1 for the single path allocation process, the total delivery route is obtained by repeatedly allocating *k* times.

#### (2) Population initialization and fitness function

After the chromosome coding is completed, an initial population containing several chromosomes is generated according to the characteristics of the problems studied. Fitness function is an important index to evaluate the quality of a chromosome. The larger the fitness value, the more likely it will be inherited to offspring. In this paper, the objective is to minimize the total routes distance, and the fitness value takes the inverse of the objective function, and the calculation is shown in formula (28).


$$fitness=\frac{1}{Z}$$ (28)

#### (3) Selection

According to the fitness value, some individuals were selected from the original population to the new population with a certain probability. The greater the fitness value, the greater the probability being selected. In this paper, stochastic universal sampling (SUS) is used to avoid monopolizing offspring due to the influence of individuals with large fitness value.

#### (4) Crossover

The crossover operator adopts Partial-Mapped Crossover (PMX). Two integers in the interval [1, n] are randomly generated to determine the positions of the two intersecting endpoints. The genes between the two endpoints of the two chromosomes are exchanged in order. Then the genes that are partially duplicated in the original chromosome are eliminated. The corresponding relationship between the exchanged parts of the two parent chromosomes is used to map and complete the chromosomes in turn.

#### (5) Variation

Exchange-mutation (EM) is used to determine mutation operator. Two integers in [1, n] interval are generated randomly, and the genes corresponding to two integers in a chromosome are exchanged.

#### (6) Reversal of evolution

In order to improve the local search ability of genetic algorithm, several successive reversal operations are used to evolve. Two integers in the interval [1, n] are randomly generated to reverse the gene at the corresponding position between two integers in a chromosome. The reversal operator is unidirectional, and only the chromosome with improved fitness after reversal can be retained, otherwise the reversal is invalid.

Algorithm 2: GA*()

1 Input: *K*, *U* = {*U*_1_, *U*_2_,⋯,*U*_*k*_}, *T* = {*T*_1_, *T*_2_,⋯,*T*_*k*_}, *population*, Maximal genetic algebra *gen_max*

2 Output: *best_dis*

3 *Z* ← 0, *gen* ← 1, *k* ← 1;

4 while *gen* < *gen_max* do

5  Traverse sequentially *population*;

6  for *k* ∈ *K* do

7   *Single path planning*();

8   for *i*, *j* ∈ *U*_*k*_ do

9    *E*_*k*_ ← *E*_*k*_ + *d*_*ij*_;

10   for *i*, *j* ∈ *T*_*k*_ do

11    *F*_*k*_ ← *F*_*k*_ + *d*_*ij*_;

12   *Z* ← *Z* + *E*_*k*_ + *F*_*k*_;

13   *k* ← *k* + 1;

14  *fitness* ← 1/*Z*;

14  best_dis ← Z

16  Select: *sus*();

17  Recombine: *pmx*();

18  Mutate: *em*();

19  *Reverse*();

20  Update *population*;

21  *Terminal optimization*();

22  if *new_min fitness* < *min fitness* then

23   *best_dis ← new_Z*;

24  *gen* ← *gen* + 1;

25 return *best_dis*;

### 4.2 Route optimization of single distribution

For the problem of single UAV and single vehicle, the objective function is to minimize the total delivery distance in this paper, the vehicle does not need to wait for the UAV to return in place, and can optimize the end of part of the joint delivery routes. When the UAV deliver for one or more nodes, the vehicle only deliver one node (this node is a stop, or include a delivery center), the two path schemes are shown in Fig 3. In order to minimize the path distance, the single distribution distance of the UAV is calculated as shown in formula (29), and the single distribution distance of the vehicle is calculated as shown in formula (30). (*E*_*k*_ *F*_*k*_) ≤ *εE*_*k*_, the scheme shown in Fig 3(a) is adopted; (*E*_*k*_ *F*_*k*_) ≥ *εE*_*k*_, the scheme shown in Fig 3(b) is adopted, and the pseudo code is shown in algorithm 3.

**Fig 3:** Terminal distribution route scheme.


Ek=∑i∈(Uk∪P)i≠j∑j∈(Uk∪P)xij,kdij∀k∈K (29)

Fk=∑i∈(Tk∪P)i≠j∑j∈(Tk∪P)εyij,kdij∀k∈K (30)

Algorithm 3: *Terminal optimization*();

1 Input: *U*_*k*_, *T*_*k*_, *E*_*k*_, *F*_*k*_, *K*

2 Output: *Z*

3 *Z* ← 0, *k* ← 1;

4 for *k* ∈ *K* do

5  if |*U*_*k*_| ≥ 1 and |*T*_*k*_| == 1 then

6   if (*E*_*k*_ *F*_*k*_) > ε*E*_*k*_ then

7    *E*_*k*_←0

8    *F*_*k*_ ← ε*E*_*k*_;

9   *T*_*k*_ ← *T*_*k*_ ⋃ *U*_*k*_;

10   *U*_*k*_ ← ∅;

11  *Z* ← *Z* + *E*_*k*_ + *F*_*k*_;

12  *k* ← *k* + 1;

13 return *Z*;

## 5 Example analysis

The heuristic algorithm designed in this paper is programmed by MATLAB r2019a and runs on a computer with Intel(R) core(TM) i7-8550u processor, 8G memory and win10 64 bit operating system. The genetic algorithm population size is 200, the selection probability is 0.9, the crossover probability is 0.9, the mutation probability is 0.05, and the maximum genetic algebra is 300. The parameter settings of the model are shown in Table 1.

**Table 1:** Parameters of the model.

Parameter	Value
Maximum payload of UAV	5
Maximum flying distance of UAV	30
Average flying speed of UAV	50
Average speed of the vehicle	50
Road impedance coefficient	1.3

### 5.1 Simulation

Considering the characteristics of mountain cities, according to the data of rc201 in Solomon case data set, we modified the cargo demand of some customer demand nodes, and added two nodes beyond the weight limit and two nodes beyond the distance limit, and generated a case in which there are 30 customer demand nodes. The information of each node is shown in Table 2. Input the data and run the program.

**Table 2:** Data of each node.

No.	X axis	Y axis	Demand	Tag	No.	X axis	Y axis	Demand	Tag
1	28	85	2	-	16	24	80	4	-
2	58	85	2	-	17	85	35	3	-
3	40	5	1	-	18	49	42	1.3	-
4	8	45	2	-	19	8	40	4	-
5	55	77	1	-	20	92	68	2	Super far node
6	55	20	1.9	-	21	85	25	1	-
7	5	5	1	Super far node	22	5	35	1	-
8	40	15	20	Overweight node	23	22	75	3	-
9	45	65	0.9	-	24	65	52	1.4	-
10	2	40	2	-	25	20	81	1	-
11	52	81	1	-	26	3	45	1	-
12	20	85	2	-	27	35	5	2	-
13	58	75	20	Overweight node	28	67	85	2	-
14	41	10	3	-	29	49	58	1	-
15	28	80	1	-	30	87	30	1	-
					31	40	50	0	Delivery center

As shown in Fig 4, the UAV can deliver multiple customer demand nodes at a single time, and at the same time, the vehicle can also deliver without waiting in place. In addition, those nodes whose demand exceeds the limit can be used as the parking spots of UAVs, while those nodes whose distance exceeds the limit can only be delivered by vehicles. The UAV and the vehicle leave the delivery center respectively, and finally the vehicle carries the UAV and returns to the delivery center at the same time. Single UAV and single vehicle carry out joint delivery, and cooperate to complete the task of all customer demand nodes. As shown in Table 3, because the customer nodes in mountain cities are scattered and relatively far away, and the UAV is limited by the maximum flight distance, and a single flight cannot go back and forth for a long distance, the customer demand nodes of vehicle delivery are more than that of UAV delivery.

**Fig 4:** Results of UAV-vehicle joint delivery.

**Table 3:** Case simulation results.

Delivery times	UAV		Vehicle	
	Route	Distance	Route	Distance
1	31 = > 18 = > 29	28.04	31 = > 29	12.04
2	-	-	29 = > 24	22.21
3	-	-	24 = > 20	40.80
4	-	-	20 = > 17	43.85
5	17 = > 30 = > 21	10.77	17 = > 21	10.00
6	-	-	21 = > 6	39.54
7	-	-	6 = > 8	20.55
8	8 = > 14 = > 23 = > 27	15.20	8 = > 27	11.18
9	-	-	27 = > 7	39.00
10	-	-	7 = > 22	39.00
11	22 = > 10 = > 26 = > 4	15.93	22 = > 19 = > 4	10.83
12	-	-	4 = > 23	43.04
13	23 = > 25 = > 12 = > 1 = > 15	23.32	23 = > 16 = > 15	9.39
14	-	-	15 = > 11	31.23
15	11 = > 2 = > 28 = > 13	29.66	11 = > 5 = > 13	8.61
16	-	-	13 = > 9	21.32
17	-	-	9 = > 31	20.55
Number of customer nodes	11		19	

In order to solve such problems, different accurate algorithms and heuristic algorithms have been designed, but the calculation time of more than 20 nodes is more than 10 minutes [13, 14]. In order to test the solution efficiency of the algorithm designed in this paper, the design algorithm (GA*) is compared with the traditional genetic algorithm (GA) and simulated annealing algorithm (SA). The programs run 30 times each. The statistical calculation results are shown in Fig 5.

**Fig 5:** Different algorithm solution results.

The three meta-heuristic algorithms can calculate the results within 1 minute, and the result box is shown in Fig 5. Because the process of decoding and updating the designed solution is complex, the variation range of the result of GA* solution is greater than GA, but less than SA. It can be seen that the convergence result of genetic algorithm is obviously better than simulated annealing algorithm in solving this problem. However, with the increase of the number of nodes, it is easy to fall into local optimization and cannot converge to the optimal value when solving this kind of problem with simple heuristic algorithm. In the figure, the minimum value and mean value of GA* solution are lower than the other two algorithms. The algorithm designed in this paper can solve good results in a short time.

### 5.2 Scene design

In order to verify the effectiveness of the model, three scenarios are designed:

1. Vehicle independent delivery: the classic TSP problem, there is no load and endurance limit for the vehicle, and considering the impact of impedance, the vehicle starts from the delivery center, and returns to the delivery center after the delivery has been done to all customer demand nodes.
2. UAV and vehicle independent delivery: multi vehicle routing problem with capacity constraints (the expansion of PDSTSP problem), vehicle and UAV are responsible for their own customer nodes, there is no cooperation between vehicle and UAV, single distribution of UAV needs to return to the delivery center to pick up and replace the power supply.
3. UAV and vehicle joint delivery: the route optimization problem proposed in this paper.

In order to minimize the delivery distance, heuristic algorithm is used to solve the three models in three scenarios. The data of 30 customer nodes in 5.1 is used, and other parameters are unchanged. Each model runs 30 times independently. Fig 6 shows the results of each run. The statistical results are shown in Table 4. The comparison of results in different scenarios is shown in Fig 6.

**Fig 6:** Running results of each scenario.

**Table 4:** Statistical results of each scenario.

Scene	Total distance					
	Max	Gap	Avg	Gap	Min	Gap
1	572.73	-	539.21	-	530.21	-
2	633.34	10.58%	556.76	3.25%	523.62	-1.24%
3	585.60	2.25%	545.94	1.25%	522.89	-1.38%

As can be seen from Fig 6, the fluctuation of scenario 1 is relatively stable, and the fluctuation amplitude of scenario 2 is the largest. Some special customer demand nodes are allocated to UAV delivery, which will result in long-distance round-trip of UAV. When the impedance is small, it will greatly increase the total delivery distance, and the fluctuation amplitude of scenario 3 is relatively stable. In Table 4, the optimal results of scenario 2 and scenario 3 using UAV delivery are less than those of scenario 1 using vehicle delivery only. The optimal solution is the UAV vehicle joint delivery of scenario 3, with an optimal value of 522.89, followed by the minimum result of scenario 2 of 523.62, compared with traditional vehicle delivery, the delivery distances of the two scenarios decrease by 1.38% and 1.24% respectively. It can be seen that adding UAV for delivery can reduce the total route distance, but because of the particularity of UAV, the route problem becomes more complex. In the heuristic algorithm, it is easy to fall into the local optimum, and resulting in some results obviously inferior to the results using only vehicle delivery, which can be seen in Fig 6.

When the delivery conditions of all customer nodes cannot not met by UAVs, the joint delivery problem is the vehicle route problem of single delivery (VRP); When the UAV can only stop at the delivery center, it becomes the UAV and the vehicle independent delivery routing problem (PDSTSP). In general, the UAV and vehicle joint delivery designed in this paper is better than the vehicle delivery and UAV vehicle independent delivery in the distribution route distance.

### 5.3 Sensitivity analysis

Due to the influence of the selected parameters on the delivery scheme, the sensitivity of the five parameters in Table 1 is analyzed for the joint delivery problem of single UAV and single vehicle in this paper. Similarly, using the node data in Table 2, except for the parameters of sensitivity analysis, the values of other parameters remain unchanged. Taking the minimum distance of the route as the goal, the design algorithm is used to solve the problem. Each group of results runs independently for 20 times, and then the minimum value is taken.

#### (1) Maximum payload and maximum flight distance of UAV

For its small size and carrying power, the UAV can load a very limited amount of goods. In addition, due to the limited battery power carried, the flight distance of UAV is small [19]. However, in a single distribution, the full load rate of UAV may be low. In order to improve the utilization efficiency of UAV, the maximum load capacity and maximum flight distance of UAV are analyzed respectively. The results under each scenario are shown in Figs 7 and 8 respectively.

**Fig 7:** Results of three scenarios under different loads.

**Fig 8:** Results of the three scenarios under different flight distances.

As can be seen from Figs 7 and 8, the vehicle delivery in scenario 1 is not affected by the maximum load and flight distance of UAV and the optimal result remains unchanged. In Fig 7, with the increase of the maximum load capacity of UAV, the number of customer nodes that UAV can delivery increases, the total route length of scenarios 2 and 3 decreases for the increase of UAV delivery nodes, however, when the maximum load of UAV increases to a certain value, affected by the delivery density of surrounding customer demand nodes, all nodes in the maximum flight distance of UAV may be delivered. Increase the load, scenario 3 can no longer reduce the total route distance. In scenario 2, due to the increase of surrounding delivery nodes, the route distance decreases, even less than scenario 3 when the load capacity is 6–8.

In Fig 8, keeping the maximum load of UAV unchanged, the results of scenario 2 change little with the increase of the maximum flight distance of UAV. Although the number of delivery nodes of UAV increases, the route distance is unreasonable when point-to-point and long distance delivery. In scenario 3, the total delivery distance increases sharply after the maximum flight distance is higher than 40. Due to different degrees of dispersion of customer demand nodes, when the flight distance of UAV is small and is not enough to delivery customer nodes, customer nodes are preferentially allocated to UAV to delivery, and the route sum of UAV and vehicle will be greater than that of vehicle separate delivery, When the maximum flight distance is increased to serve multiple customer nodes in a single distribution, the joint delivery of UAV and vehicle can effectively reduce the total delivery route. However, limited by the maximum load capacity of the UAV, continuing to increase the maximum flight distance will make the UAV deliver to customer nodes at a long distance, and the round-trip stop will greatly increase the total route length.

#### (2) Average flight speed of UAV and average driving speed of vehicle

The vehicle must arrive at the stop before the UAV arrives. Under the condition of meeting the maximum flight distance of the UAV, the average flight speed of the UAV and the average driving speed of the vehicle determine the maximum distribution distance they can travel [24]. Under the different combination of UAV and vehicle speed, the efficiency of delivery is different. The combination of UAV and vehicle at different speed ratios is shown in Table 5, and the results are shown in Fig 8.

**Table 5:** Combinations of UAV and vehicles at different speeds.

Average flying speed of the UAV	Average speed of the vehicle	Speed ratio
40	100	1:2.5
50	100	1:2
50	75	1:1.5
50	50	1:1
75	50	1.5:1
100	50	2:1
100	40	2.5:1

As shown in Fig 9, when the speed of UAV is far less than the speed of vehicle, the vehicle cannot arrive before the UAV arrives at the stop, most customer nodes will be allocated to vehicles for delivery, and the UAV can only deliver a very small number of customer demand nodes. With the increase of UAV flight speed, UAV can deliver more customer demand nodes. However, due to the limited customer demand nodes, the total route length of joint delivery is not necessarily less than the total route length of vehicle single delivery. When the UAV flight speed exceeds the vehicle speed and the UAV can complete the delivery task of multiple customer demand nodes, the total delivery distance decreases significantly. However, when the UAV’s flight speed exceeds twice the vehicle’s speed, the total route length will not be reduced due to the maximum load and flight distance of UAV.

**Fig 9:** Results of three scenarios at different speed ratios.

#### (3) Impedance coefficient

The roads in mountainous cities are circuitous and rugged, and there are even no roads in some places, which is very inconvenient for vehicles to get in and out. When vehicles are distributed in different environments, they are vulnerable to road conditions. The more complex the terrain is, the higher the impedance coefficient is. Therefore, the delivery route of vehicles needs to be adjusted appropriately, and the route of UAV will also be affected by the driving route of vehicles.

The delivery route results under different impedance coefficients are shown in Fig 10. The total delivery distance of the three scenarios increases almost linearly with the increase of impedance coefficient. Compared with traditional delivery, the biggest advantage of UAV delivery in delivery distance is that it cannot be limited by terrain. When the road impedance coefficient exceeds 1.7, scene 2 and scene 3 with UAV delivery are significantly better than scene 1 without UAV delivery. With the increase of impedance coefficient, the advantage of joint delivery is more obvious.

**Fig 10:** Results under different impedance coefficients.

In general, the joint delivery efficiency of UAV and vehicle is limited by the above parameters. When the number of customers that can be delivered by UAV is sufficient, increasing the maximum carrying capacity and maximum flight distance of UAV, as well as increasing the relative speed of UAV and vehicle can effectively reduce the length of the total delivery route. The number of customer points that can be distributed by UAV in a single time will increase, and the overall delivery efficiency will increase. However, when it is raised to a certain extent, the distribution of surrounding customer points will have an impact on the delivery results UAVs and vehicles may have long-distance round-trip, increasing the delivery distance.

## 6 Conclusion

Based on the logistics distribution in mountainous cities, this paper considers the delivery characteristics of UAVs and the impact of terrain environment, and proposes a UAV-vehicle joint delivery model. Aiming at the problem of single-UAV and single-vehicle joint delivery, after the UAV is launched from the vehicle, it can deliver multiple customer demand points. A three-step route distribution method is designed to mark special points, single path planning, and overall route optimization. In the presence of impedance, with the minimum total delivery distance as the objective function, the genetic algorithm with end optimization is used to solve the proposed problem through case simulation. The results show that the proposed joint delivery model can improve the efficiency of delivery, reduce the length of the total delivery route and can solve the logistics distribution problems in mountain cities.

In the future, UAV technology will be further improved, the load capacity and flight distance of UAV will be strengthened, its advantages of low cost and ignoring terrain will be more prominent, and faster, more energy-saving and efficient logistics distribution will become a trend. In the next step, we can consider increasing the number of vehicles, expanding the joint delivery to multi UAV and multi vehicle scenarios, and increasing the time window limit of customer points; More uncertain factors (weather influence, signal interference, etc.) can also be added to enrich the application scenarios of logistics distribution. After the UAV related laws and regulations are perfected, it can be expanded to more urban areas for logistics distribution.

## Supporting information

S1 Data (XLSX)
